# Development and Validation of a Novel Model for Predicting the 5-Year Risk of Type 2 Diabetes in Patients with Hypertension: A Retrospective Cohort Study

**DOI:** 10.1155/2020/9108216

**Published:** 2020-09-27

**Authors:** Xintian Cai, Qing Zhu, Ting Wu, Bin Zhu, Xiayire Aierken, Ayguzal Ahmat, Nanfang Li

**Affiliations:** Hypertension Center of People's Hospital of Xinjiang Uygur Autonomous Region; Xinjiang Hypertension Institute; National Health Committee Key Laboratory of Hypertension Clinical Research, Urumqi, Xinjiang 830001, China

## Abstract

**Background:**

Hypertension is now common in China. Patients with hypertension and type 2 diabetes are prone to severe cardiovascular complications and poor prognosis. Therefore, this study is aimed at establishing an effective risk prediction model to provide early prediction of the risk of new-onset diabetes for patients with a history of hypertension.

**Methods:**

A LASSO regression model was used to select potentially relevant features. Univariate and multivariate Cox regression analyses were used to determine independent predictors. Based on the results of multivariate analysis, a nomogram of the 5-year incidence of T2D in patients with hypertension in mainland China was established. The discriminative capacity was assessed by Harrell's *C*-index, AUC value, calibration plot, and clinical utility.

**Results:**

After random sampling, 1273 and 415 patients with hypertension were included in the derivation and validation cohorts, respectively. The prediction model included age, body mass index, FPG, and TC as predictors. In the derivation cohort, the AUC value and *C*-index of the prediction model are 0.878 (95% CI, 0.861-0.895) and 0.862 (95% CI, 0.830-0.894), respectively. In the validation cohort, the AUC value and *C*-index of the prediction model were 0.855 (95% CI, 0.836-0.874) and 0.841 (95% CI, 0.817-0.865), respectively. The calibration plots demonstrated good agreement between the estimated probability and the actual observation. Decision curve analysis shows that nomograms are clinically useful.

**Conclusion:**

Our nomogram can be used as a simple, affordable, reasonable, and widely implemented tool to predict the 5-year T2D risk of hypertension patients in mainland China. This application helps timely intervention to reduce the incidence of T2D in patients with hypertension in mainland China.

## 1. Introduction

Type 2 diabetes (T2D) is a form of hyperglycemia caused by insulin resistance and related insulin deficiency, accounting for 90%-95% of all diabetes [1]. The growing burden of T2D has become the focus of global public health attention in the 21st century [2]. Previously, T2D was the most common in the rich “western” developed countries [3]. But at present, T2D has become an epidemic in developing countries [4]. China is among the most populous countries in the world, and the country with the most diabetes cases in the world, with an estimated 120.9 million adults suffering from diabetes [5]. T2D patients have to bear high medical expenses every year. It is estimated that the global medical expenditure for T2D in 2017 was approximately $850 billion [6]. In addition, T2D can cause a variety of complications, such as diabetic nephropathy, cardiovascular and cerebrovascular diseases, and diabetic retinopathy [3]. There are numerous causes of T2D. Although the specific reasons are not clear, a large number of studies have pointed out that T2D may be related to lifestyle, genetic susceptibility, and environmental factors [4].

High blood pressure is the single only risk factor responsible for the global burden of disease, and 9.4 million people worldwide die of hypertension every year [7]. It is pointed out that hypertension and T2D often coexist, and about 70% of T2D patients also have hypertension [8]. Patients with a history of hypertension are nearly 2.5 times more likely to develop T2D than normal people [9]. Compared with patients with hypertension or T2D alone, patients with hypertension and T2D have an increased risk of all-cause and cardiovascular death [10]. Analysis of the Framingham cohort showed that patients with elevated blood pressure at the time of T2D diagnosis had higher rates of cardiovascular disease (CVD) and all-cause mortality than patients without T2D [11].

Due to the greatly increased prevalence of diabetes in patients with a history of hypertension, it has caused huge economic costs and serious complications. Therefore, the purpose of this study is to establish an effective risk prediction model, which can provide an early prediction for the risk of new-onset diabetes in patients with a history of hypertension, provide timely intervention measures to prevent or delay the occurrence of T2D, and ultimately reduce the adverse cardiovascular prognosis of such patients.

## 2. Methods

### 2.1. Study Population and Follow-Up Evaluation

The data for this study can be for download from a shared database called the Dryad Digital Repository (http://www.datadryad.org/), with an identifier of 10.5061/dryad.ft8750v. The database is funded by the National Science Foundation of the United States. It is a place to store high-quality data resources to discover, reuse, and cite data behind scientific publications. Its goal is to form an academic exchange system with academic groups, publishing, research and education institutions, funding agencies, and other stakeholders to coordinate, maintain, and promote the protection and reuse of basic data in academic literature. The original data was provided by Chen et al. [12]. The raw data was extracted from a computer database established by Rich Healthcare Group, which includes all medical records of participants who underwent medical examinations in 32 locations and 11 cities in China from 2010 to 2016. All participants were older than 20 years of age and had at least two visits between 2010 and 2016 (*n* = 685277). They are not included in the baseline if any of the following conditions are met: participants have no available weight and height measurements, no available gender information, no available blood pressure values, missing questionnaire data (including smoking status, drinking status, and family history of diabetes), extreme body mass index (BMI) values (<15 kg/m^2^ or >55 kg/m^2^), no fasting plasma glucose value (FPG), no serum triglycerides (TG), no total cholesterol (TC), no low-density lipoprotein cholesterol (LDL-C), no alanine aminotransferase (ALT), no aspartate aminotransferase (AST), no blood urea nitrogen (BUN), no creatinine clearance (CCR), and no high-density lipoprotein cholesterol (HDL-C). We further excluded subjects who were followed up for less than 2 years; baseline subjects diagnosed with diabetes, coronary heart disease, heart failure, and valvular heart disease; and subjects with uncertain diabetes status at follow-up. A total of 1688 baseline patients with complete information and history of hypertension but no diabetes were obtained. All subjects underwent at least two follow-up visits at intervals of ≥2 years between 2010 and 2016. We downloaded the raw data and performed a secondary analysis. In order to establish and validate the prediction model, a simple random method was used to randomly select 75% of the patients as the derivation cohort and the remaining 25% as the validation cohort.

### 2.2. Variable Measurement

Well-trained staff obtained detailed demographic characteristics, lifestyle, past medical history, and family history of chronic diseases by conducting detailed questionnaires on each subject. Height, weight, and blood pressure were measured by trained staff. Using a height and weight scale to measure height to the nearest 0.1 cm and weight to the nearest 0.1 kg. The scale was calibrated before use, with participants wearing light, shoeless clothing. Body mass index (BMI) was calculated based on body weight (kg)/height^2^ (m^2^). After at least 5 minutes of rest, blood pressure was measured by a standard mercury sphygmomanometer. Prior to each visit, the respondents fasted for at least 10 hours overnight. Venous blood samples were collected after fasting and processed within 2 hours. Serum TG, TC, LDL-C, HDL-C, ALT, AST, BUN, and CCR were measured on Beckman 5800. Plasma glucose levels were measured on an automatic analyzer (Beckman 5800) by the glucose oxidase method.

### 2.3. Data Collection

The variables for each case were extracted from the raw data as follows: age, gender, fasting blood glucose (FPG), BMI, systolic blood pressure (SBP), diastolic blood pressure (DBP), TC, TG, HDL-C, LDL-C, ALT, AST, BUN, CCR, smoking status, drinking status, family history of diabetes, years of follow-up, and eventual diagnosis of diabetes. Incomplete records were excluded.

### 2.4. Definitions

Hypertension is defined as SBP ≥ 140 mmHg or/and DBP ≥ 90 mmHg. Smoking status can be divided into three categories: never smoker, ever smoker, or now smoker. Drinking status is divided into three categories: never drinking, ever drinking, or now drinking. The family history of diabetes was divided into the positive and negative groups. During the follow-up period, FPG ≥ 7.00 mmol/L or/and self-reported diabetes can be diagnosed as sudden diabetes. Patients were checked at the time of diagnosis of diabetes or the last visit, whichever came first.

### 2.5. Feature Selection

The least absolute shrinkage and selection operator (LASSO) logistic regression algorithm is a punitive regression method. It estimates the regression coefficient by maximizing the logarithmic likelihood function and limits the sum of the absolute values of the regression coefficients [13]. The regression coefficient estimated by LASSO is very sparse, and many components are exactly 0 [14]. Therefore, the LASSO automatically removes unnecessary covariates. The LASSO logistic regression algorithm can be used for regression analysis of high-dimensional data [15]. In this study, the LASSO logistic regression algorithm was used to select the most important prediction features in the derivation data set [16]. All category variables are converted to dummy variables. The state of T2D was used as a dependent variable. Cross-validation was used to determine the appropriate adjustment parameter (*λ*) for LASSO logistic regression [13, 15].

### 2.6. Statistical Analysis

The continuous variables with normal distribution are expressed as mean ± standard deviation, and category variables are expressed as frequency (percentage). In the derivation cohort, the multivariate Cox proportional risk regression analysis was used to further evaluate the factors with statistical significance in the univariate analysis. The features selected in the derivation data set using the LASSO algorithm were utilized to construct a nomogram through a multivariate Cox regression analysis. A nomogram was utilized to show the risk prediction model of new-onset T2D in patients with hypertension. The prediction model was evaluated from three aspects: discrimination ability, calibration ability, and clinical effectiveness. The nomogram was verified internally in the derivation cohort and externally in the validation cohort. Harrell's *C*-statistical consistency index (*C*-index) was applied to the evaluation of nomogram identification [17]. The *C*-index value ranges from 0.5 to 1.0, where 0.5 represents random chance and 1.0 represents exactly the same. In general, *C*‐index > 0.7 was considered to have excellent discrimination [18]. The area under the ROC curve (AUC) was used to evaluate the prediction discrimination of the nomogram. In the regression model, AUC value was similar to *C*-index, and AUC value > 0.7 was considered to have better discrimination ability. The calibration capability was evaluated through the calibration chart and the Hosmer–Lemeshow test [19]. The bootstrap method with 1000 resamples was applied to measure the *C*-index, AUC value, and calibration curve [20]. A decision curve analysis (DCA) was used to evaluate the clinical usefulness of the nomogram based on its net benefits at different threshold probabilities in the validation cohort. All tests were two-tailed, and a *P* value of < 0.05 was considered statistically significant. All statistical analyses were carried out using R software (http://www.r-project.org/) with the R base package.

## 3. Results

### 3.1. Characteristics of Study Population

A total of 1688 patients participated in our study, and 103 of them developed diabetes. The median follow-up time for all participants in this study was 3.0 years (range: 2.0-5.7 years). Eligible participants were randomly split into a derivation cohort (*n* = 1273) and a validation cohort (*n* = 415). The ages of the derivation group and the validation group were 48.09 ± 12.91 years and 48.97 ± 13.54 years, respectively. The BMI of the derivation group and the validation group were 25.57 ± 3.29 kg/m^2^ and 25.55 ± 3.36 kg/m^2^, respectively. The FPG of the derivation group and the validation group were 5.23 ± 0.67 mmol/L and 5.25 ± 0.68 mmol/L, respectively. The average follow-up time of the derivation and the validation groups was 1078 days and 1087 days, respectively. There were 81 and 22 T2D cases in the derivation and validation cohorts, respectively. There were no statistical differences between the two groups in FPG, follow-up time, incidence of T2D, age, gender, BMI, TC, TG, LDL-C, ALT, AST, BUN, CCR, smoking status, drinking status, and family history. The baseline characteristics of the derivation and validation cohorts are set out in Table 1.

### 3.2. Feature Selection

The LASSO logistic regression method was employed to select the most significant prediction features in the prediction model. In this study, feature selection was carried out based on the derivation dataset. In total, 20 features were used in LASSO logistic regression. Moreover, eight features with nonzero coefficients were selected by the LASSO logistic regression algorithm with an optimal *λ* of 0.0212 (Figures 1(a) and 1(b)). These eight features include Aage, BMI, FPG, TC, HDL-C, smoking status, drinking status, and family history.

### 3.3. Independent Risk Factors in the Derivation Cohort

In patients with a history of hypertension, the variables identified as predictors of incident T2D are listed in Table 2. In the derivation cohort, univariate Cox regression analysis showed that age, BMI, FPG, TC, TG, HDL-C, CCR, smoking status, drinking status, and family history were significant risk factors for T2D in addition to gender, LDL-C, ALT,AST, and BUN. Multivariate Cox regression analysis showed that age, BMI, FPG, and TC are independent risk predictors for the development of T2D in patients with a history of hypertension, which can be further used to establish a nomogram.

### 3.4. Nomogram Construction and Performance Assessment

As shown in Figure 2, the nomogram was drawn to provide a quantitative and convenient tool to predict the 5-year incidence of T2D in patients with hypertension by using age, BMI, FBG, and TC in the derivation cohort. To assess the 5-year risk of T2D in a hypertensive patient, the value of the hypertensive patient was located on each variable axis. A vertical line was drawn from the value to the vertex scale to the number of points at which the variable value is specified. Then, points from each variable value are summed. The sum was located on the total submark and projected vertically on the bottom axis to obtain the individualized risk of T2D in this hypertensive patient for 5 years. ROC curves are shown in Figures 3(a) and 3(b). The obtained model was validated internally by bootstrap method with 1000 resamples. In the derivation cohort, the AUC value and the *C*-index were 0.793 (95% CI, 0.776-0.810) and 0.802 (95% CI, 0.770-0.834), respectively, with good discrimination ability. Similarly, in the validation cohort, the AUC value and the *C*-index of the model were 0.779 (95% CI, 0.756-0.802) and 0.781 (95% CI, 0.757-0.815), respectively, which have better prediction effect. A calibration plot and Hosmer–Lemeshow tests were utilized to calibrate the prediction model. From the calibration curve, the prediction model fits well with the validation cohort. The Hosmer–Lemeshow tests show that the predicted probability is highly consistent with the actual probability (*P* = 0.285 for the derivation cohort, Figure 4(a); *P* = 0.321 for validation cohort, Figure 4(b)). DCA was used to evaluate the clinical application value of the prediction model. From the perspective of the decision curve, the net benefit of the prediction model and the internal validation cohort were significantly higher than those of the two extreme cases where everyone was treated (Figure 5).

### 3.5. Clinical Application of the Nomogram

Hereby, we took 2 patients with hypertension as examples of the application of the nomogram. The first patient was 65 years old (15 points). The levels of BMI, FPG, and TC were 38 kg/m^2^ (36 points), 6.5 mmol/L (89 points), and 10 mmol/L (28 points), respectively. The calculated nomogram score is 168 points, and the 5-year risk probability of T2D in hypertensive patients exceeds 0.9. This patient has a high risk of developing T2D in 5 years. The second patient was 50 years old (10 points). The levels of BMI, FPG, and TC were 20 kg/m^2^ (7 points), 4 mmol/L (33 points), and 10 mmol/L (28 points). The calculated nomogram score was 78, and the 5-year risk probability of T2D in patients with hypertension was less than 0.1. The second patient had a very low risk of T2D at 5 years.

## 4. Discussion

With the development of the economy and the improvement of people's living standards, T2D is on the rise worldwide, which is thought to be the third largest disease that threatens human health, next to cancer and cardiovascular disease [21]. T2D and its complications are one of the major economic burdens in the present era [22]. China has the largest number of patients with diabetes in the world. According to the International Diabetes Federation, the annual cost of diabetes in China is $ 25 billion [23]. It is estimated that these costs will continue to increase and will exceed $ 47 billion by 2030 [24]. A large number of studies have shown that hypertension is closely related to impaired glucose tolerance [25]. T2D is more common in patients with hypertension than in patients without a history of hypertension. The coexistence of DM and hypertension significantly increase the risk for coronary heart disease, left ventricular hypertrophy, congestive heart failure, and stroke compared to either condition alone [10]. In addition, both hypertension and DM are present in all prediction models for the occurrence of stroke in patients with atrial fibrillation [26]. Microvascular complications are also more common in patients with coexistent hypertension and DM, and both retinopathy and nephropathy are more prevalent in patients with DM and hypertension [10]. Therefore, primary prevention and timely intervention are the keys to prevent or delay the onset of T2D in patients with hypertension [11]. Early detection of people at high risk for diabetes is critical to reducing morbidity, which led us to this study.

In this community-based cohort study, we developed a quantifiable and simple nomogram to predict the 5-year T2D risk of hypertension patients in mainland China. In the derivation and validation cohorts, our model shows higher prediction accuracy, relatively high *C*-index, and excellent calibration curve consistency. As far as we know, this study is the first nomogram to estimate the risk of type 2 diabetes in Chinese mainland hypertension patients using continuous values rather than segmented values. In addition, the nomogram will be of great practical value because of their easily obtained parameters. In this study, we developed a nomogram based on a large-scale multicenter population of China. Although it has been reported that more than 40 T2D risk prediction models have been established among different populations, there are few risk prediction models based on the East Asian race, especially the Chinese population [27–30]. Taking into account the genetic and environmental differences (i.e., economic level, diet, climate, and lifestyle), the intensity or distribution of T2D risk factors varies among different populations, complex mathematical formulas, and the lack of simple and intuitive tools to facilitate the use of these predictive risk models [14]. Therefore, few models are currently used clinical practice. Our study is the first nomogram to predict the 5-year incidence of T2D in hypertensive patients in mainland China. Nomogram is a graphical representation of a complex mathematical formula, which is widely used in the study of tumor prognosis [31, 32]. However, a few types of research have focused on developing this easy-to-use T2D risk prediction tool. The nomogram can generate individual T2D probability by integrating various risk prediction factors, which can meet our needs for visualization tools and meet our progress towards personalized prevention [33]. Compared with traditional mathematical formulas, through the user-friendly digital interface, higher accuracy, and easier to understand risk prediction, rapid calculation of the nomogram can seamlessly integrate risk assessment into clinical decision-making [34]. Using these simple, fast, cheap, noninvasive tools, we hope to be able to effectively identify individuals with a high risk of 5-year T2D in patients with hypertension. Medical interventions, lifestyle changes, diagnostic management, and treatment then can be initiated, and ultimately the patient's prognosis can be improved.

Our prediction models include age, BMI, FBG, and TC. These variables identified as risk factors for T2D were consistent with previous studies. Multiple studies have found that dyslipidemia, obesity, and T2D usually coexist in individuals and share common pathological mechanisms (metabolic disorders, insulin resistance, inflammation, and changes in the intestinal flora) [35–37]. Therefore, the application of these parameters in the model is well founded. T2D usually occurs in adults and is more common in the elderly. Numerous studies have proven that advanced age is an unchangeable risk factor for the manifestation of diabetes [3, 38]. Aging *β*-cells may exhibit lower glucose responsiveness and glucose sensitivity, leading to hyperglycemia and T2D [39]. The epigenetic changes caused by aging may affect islet gene expression and insulin secretion [40]. Davegårdh et al. [41] found that age-related changes in pancreatic islet DNA methylation can increase insulin resistance, cause impaired *β*-cell function, and induce T2D. Impaired FBG is one of the diagnostic criteria for diabetes. Studies have shown that hemoglobin A1c, FBG, and 2hPG can predict diabetes, but the detection reliability of hemoglobin A1c and FBG is better than 2hPG [42]. In addition, compared with A1c hemoglobin, the feasibility and applicability of FBG detection in low-resource settings are more prominent [43]. In our predictive model, BMI was one of the main aspects of all diabetic risk factor scores. It is well known that T2D is usually associated with overweight and obese individuals [44, 45]. Obesity, especially long-lasting and visceral obesity, is the cornerstone of T2D pathogenesis [46]. According to gender and ethnicity, the incidence rate of BMI in patients with T2D ranges from 50% to 90% was 25 kg/m^2^, and the incidence of T2D in elderly obese patients was higher [47]. It is worth noting that even if BMI is less than 25 kg/m^2^, the relative risk of diabetes in adults seems to increase, and it increases exponentially with BMI [47]. The pathophysiological pathways behind this association are complex and progressive, leading to the development of insulin resistance and secondary impairment of *β*-cell function [44, 46, 47]. Obesity-induced metabolic disorders, adipose organ dysfunction, and changes in fat metabolic processes play a fundamental role in insulin resistance [44]. Excess energy induces insulin resistance by inhibiting adenosine monophosphate-activated protein kinase signaling pathways in obese patients [44, 48]. According to previous studies, dyslipidemia is a well-known risk factor for T2D [49]. Similar to those reports, patients with TC abnormalities had higher T2D risk scores on the nomogram. The underlying pathophysiology of dyslipidemia leading to insulin resistance is complex and has not been well understood [36]. At present, some studies have pointed out that TC itself may directly lead to disorders of glucose metabolism [37, 50]. TC can also increase insulin secretion by protecting *β*-cells from cholesterol-induced *β*-cell dysfunction, stress-induced apoptosis, and islet inflammation [46, 47]. The higher level of TC may exacerbate abnormal glucose homeostasis. In contrast, oxidized low-density lipoprotein can inhibit molecular insulin secretion and even cause *β*-cell apoptosis [39, 40].

In this study, we established a nomogram model of 5-year T2D incidence of hypertension patients in mainland China by using parameters that can be collected in the general health care settings. This will have a major impact on the clinic and society, especially for residents in mainland China, where OGTT is not easily accessible. Our nomogram provides a quantitative way to distinguish the high-risk group of T2D in patients with hypertension who must focus on their own physical condition and follow advanced intervention strategies (e.g., appropriate drug intervention, lifestyle intervention, and/or surgical operation) to prevent or at least delay the development of T2D in patients with hypertension. At the same time, for low-risk T2D populations, no further screening of T2D is needed, which can increase the cost-effectiveness of T2D screening. This simple risk assessment tool can be accepted by the medical staff and nonprofessionals.

Although our nomograms performed well in both the derivation and validation cohorts, there are still some limitations in this study. First, all participants are from China. Therefore, the result may not apply to other countries. Second, although our analysis includes a wide range of potential predictors, there are other factors that cannot be measured, such as insulin secretion, which leads to the limited predictive power of the model. Third, the nomogram is based on a retrospective cohort study in which individuals with incomplete data are excluded, which may lead to selection bias. Therefore, prospective studies are needed to further validate our results. Fourth, although the genomic classifier is considered a promising predictive tool, this study did not consider genomic characteristics. Fifth, the lack of treatment data for participants in the study may interfere with the development of diabetes. Sixth, failure to perform HbA1c and oral glucose tolerance tests may mask diabetes events at baseline or during follow-up. Despite these limitations, the study was the first large cohort study in mainland China to predict 5-year T2D incidence in patients with hypertension.

## 5. Conclusion

In summary, we have established a nomogram based on four risk factors, including FBG, age, BMI, and TG, to determine the population with high T2D risk in patients with hypertension in mainland China. Our nomogram can be used as a simple, affordable, reasonable, and widely implemented tool to predict the 5-year T2D risk of hypertension patients in mainland China. This application helps timely intervention to reduce the incidence of T2D in patients with hypertension in mainland China.

## Figures and Tables

**Figure 1:** Feature selection using least absolute shrinkage and selection operator (LASSO) logistic regression. (a) Tuning parameter (*λ*) selection in the LASSO logistic regression performed using 10-fold cross-validation via the minimum criteria. The binomial deviance was plotted versus log(*λ*). Dotted vertical lines were drawn at the optimal *λ* based on the minimum criteria and 1 standard error for the minimum criteria, and the optimal *λ* was 0.0212. (b) The LASSO logistic regression algorithm was used to screen out 8 features with nonzero coefficients out of 20 features. A coefficient profile plot is produced versus the log(*λ*). LASSO: least absolute shrinkage and selection operator.

**Figure 2:** Nomogram to predict the 5-year risk of T2D in Chinese patients with hypertension. ^∗^Instructions: to estimate an individual's 5-year risk of T2D in a patient with hypertension and determine the value on each variable axis. Draw a vertical line from the value to the top points scale to determine how many points are assigned to the variable value.. Then, the points from each variable value are summed. Locate the sum on the total points scale and project it vertically on the bottom axis to obtain a personalized 5-year T2D risk.

**Figure 3:** The ROC curves of the nomogram from the derivation cohort (a) and the validation cohort (b). ROC: receiver operating characteristics curves. ^∗^Using bootstrap resampling (times = 1000).

**Figure 4:** Calibration plots of the nomogram. The shadow line represents the perfect prediction of an ideal model, and the dashed lines represent the performance of the derivation cohort (a) and the validation cohort (b).

**Figure 5:** The decision curve analysis (DCA) for the nomogram. Area within the red solid line, the grey solid line, and the black solid line represents the net beneft. The red solid line represents the nomogram. The black solid line indicates that all samples are negative and all were not treated. The grey solid line indicates that all samples were positive and were treated.

**Table 1:** Baseline characteristics of derivation and validation cohorts.

Characteristic	Derivation cohort (*n* = 1273)	Validation cohort (*n* = 415)	*P* value
Age (mean ± SD) (years)	48.09 ± 12.91	48.97 ± 13.54	0.232
BMI (mean ± SD) (kg/m^2^)	25.57 ± 3.29	25.55 ± 3.36	0.898
FPG (mean ± SD) (mmol/L)	5.23 ± 0.67	5.25 ± 0.68	0.623
TC (mean ± SD) (mmol/L)	4.97 ± 0.90	5.04 ± 0.88	0.159
TG (mean ± SD) (mmol/L)	1.92 ± 1.32	1.94 ± 1.33	0.774
HDL-C (mean ± SD) (mmol/L)	1.32 ± 0.29	1.28 ± 0.28	0.011
LDL-C (mean ± SD) (mmol/L)	2.86 ± 0.68	2.90 ± 0.69	0.263
ALT (mean ± SD) (mmol/L)	31.39 ± 23.75	32.25 ± 23.49	0.524
AST (mean ± SD) (mmol/L)	27.49 ± 12.31	28.02 ± 10.88	0.429
BUN (mean ± SD) (mmol/L)	4.92 ± 1.18	4.93 ± 1.22	0.936
CCR (mean ± SD) (mmol/L)	76.22 ± 14.99	75.72 ± 14.62	0.551
Follow-up (mean ± SD) (days)	1078.09 ± 320.10	1087.86 ± 324.96	0.591
Gender (*n*, %)			0.707
Male	995 (78.16%)	328 (79.04%)	
Female	278 (21.84%)	87 (20.96%)	
Smoking status (*n*, %)			0.173
Current	335 (26.32%)	108 (26.02%)	
Ever	72 (5.66%)	14 (3.37%)	
Never	866 (68.03%)	293 (70.60%)	
Drinking status (*n*, %)			0.896
Current	88 (6.91%)	26 (6.27%)	
Ever	265 (20.82%)	88 (21.20%)	
Never	920 (72.27%)	301 (72.53%)	
Family history (*n*, %)			0.486
No	1187 (93.24%)	391 (94.22%)	
Yes	86 (6.76%)	24 (5.78%)	
Incident T2D (*n*, %)			0.433
No	1192 (93.64%)	393 (94.70%)	
Yes	81 (6.36%)	22 (5.30%)	

Data are shown as means + SD or no. (%). BMI: body mass index; FBG: fasting blood glucose; TC: total cholesterol; TG: triglycerides; LDL-C: low-density lipoprotein cholesterol; HDL-C: high-density lipoprotein cholesterol; ALT: alanine aminotransferase; AST: aspartate aminotransferase; BUN: blood urea nitrogen; CCR: creatinine clearance; T2D: type 2 diabetes.

**Table 2:** T2D risk prediction in patients with hypertension based on Cox proportional risk regression model.

	Univariate analysis	*P* value	Multivariate analysis	*P* value
	OR (95% CI)		OR (95% CI)	
Age	1.04 (1.03, 1.06)	<0.0001	1.04 (1.02, 1.06)	0.0009
Gender				
Male	Reference			
Female	0.47 (0.25, 0.89)	NS		
BMI	1.13 (1.07, 1.20)	<0.0001	1.14 (1.05, 1.23)	0.0016
FPG	6.60 (4.95, 8.81)	<0.0001	6.21 (4.28, 8.99)	<0.0001
TC	1.28 (1.04, 1.57)	0.0203	1.26 (1.07, 1.53)	0.0188
TG	1.29 (1.20, 1.39)	<0.0001	1.05 (0.86, 1.28)	NS
HDL-C	0.29 (0.15, 0.57)	0.0003	0.93 (0.33, 2.57)	NS
LDL-C	1.17 (0.85, 1.60)	NS		
ALT	1.00 (1.00, 1.01)	NS		
AST	1.01 (1.00, 1.02)	NS		
BUN	1.13 (0.94, 1.36)	NS		
CCR	0.99 (0.97, 1.00)	0.0458	1.00 (0.98, 1.02)	NS
Smoking status				
Current	Reference		Reference	
Ever	0.62 (0.27, 1.47)	NS	0.49 (0.20, 1.18)	NS
Never	0.32 (0.21, 0.51)	<0.0001	0.95 (0.44, 2.06)	NS
Drinking status				
Current	Reference		Reference	
Ever	0.17 (0.10, 0.29)	<0.0001	0.49 (0.20, 1.18)	NS
Never	0.16 (0.08, 0.32)	<0.0001	0.95 (0.44, 2.06)	NS
Family history				
No	Reference		Reference	
Yes	3.79 (2.33, 6.15)	<0.0001	1.63 (0.82, 3.23)	NS

T2D: type 2 diabetes; BMI: body mass index; FBG: fasting blood glucose; TC: total cholesterol; TG: triglycerides; LDL-C: low-density lipoprotein cholesterol; HDL-C: high-density lipoprotein cholesterol; ALT: alanine aminotransferase; AST: aspartate aminotransferase; BUN: blood urea nitrogen; CCR: creatinine clearance; OR: odds ratio; CI: confidence interval; NS: no significance.

## Data Availability

All datasets generated and/or analyzed during the present study are included in this published article and available in Dryad Digital Repository (http://www.datadryad.org/).
